# Using the Intelligent System to Improve the Delivered Adequacy of Dialysis by Preventing Intradialytic Complications

**DOI:** 10.1155/2022/8160269

**Published:** 2022-06-23

**Authors:** Mohammad Karimi, Daryoosh Dideban, Hadi Heidari

**Affiliations:** ^1^Department of Electrical and Computer Engineering, University of Kashan, Kashan, Iran; ^2^James Watt School of Engineering, University of Glasgow, Glasgow G12 8QQ, UK

## Abstract

Acute kidney failure patients while detoxificated by hemodialysis (HD) mostly or continuously faced regular problems such as low blood pressure (hypotension), muscle cramps, nausea, or vomiting. Higher intradialytic symptom leads to low-quality HD treatment. Although more known therapeutic interventions are used to relieve the HD side effects, this study was designed to investigate how intelligent systems can make highly beneficial alterations in dialysis facilities and equipment to ease intradialytic complications and help the staff deliver high-quality treatment. A search was performed among relevant research articles based on nonpharmacological intervention methods considered to prevent adverse effects of renal replacement therapy until 2020 in the PubMed databases using the terms “intradialytic complications,” “intradialytic complication interventions,” “nonpharmacological interventions,” “intradialytic exercises,” and “adequacy calculation methods.” Studies included the prevalence of intradialytic complications, different strategies with the aim of preventing complications, the outcome of intradialytic exercises on dialysis symptoms, and dialysis dose calculation methods. The results showed the incidence of hypotension varying between 5% and 30%, fatigue, muscular cramps, and vomiting as the most common complications during dialysis, which greatly affect the outcome of HD sessions. To prevent hypotension, ultrafiltration profiling, sodium modeling, low dialysate temperature, and changing the position to Trendelenburg are some strategies. Urea reduction ratio (URR), formal urea kinetic modeling (FUKM), formal single-pool urea kinetics, and online clearance monitoring (OCM) are methods for calculating the delivered dose of dialysis in which OCM is a low-cost and accessible way to monitor regularly the quality of dialysis delivered. Integration of the chair and HD machine which is in direct contact with the patient provides an intelligent system that improves the management of the dialysis session to enhance the quality of healthcare service.

## 1. Introduction

At present, HD is a well-recognized treatment procedure that improves the quality of renal replacement therapy in end-stage renal disease (ESRD) patients [1]. HD treatment is arranged to preserve the patient's blood pressure in the proper range and remove the waste products from blood to maintain essential minerals such as potassium and sodium. HD treatment commences before the kidneys fail to the point that the progression of the disease will threaten the patient's life. The prevalence of kidney failure has become more progressive because of some commonly diagnosed reasons such as hypertension, diabetes, and kidney inflammation [2]. Therefore, more people who underwent HD therapeutic with kidney failure have a variety of health problems. Although HD treatment optimizes the patient's life expectancy, it is not satisfactory in comparison to the general population. While HD machines act as kidneys in body fluid and blood purification, the patient may experience some of the side effects such as low blood pressure (hypotension), muscle cramps, sleep problems, and anemia; however, not everyone experiences all of these issues. Hypotension is the most common side effect during dialysis, especially in older people who need and occupy a lot of staff time in the centers. This common issue mostly appeared with other complications such as muscle cramps, shortness of breathing, and vomiting. It is important to note that higher intradialytic symptoms result in poor outcomes, including decreased quality of life, decreased dialysis dose, depression, and mortality [3, 4]. Nonexperimental studies have endorsed the fact that high-quality HD therapy in patients with ESRD can mitigate the development or severity of complications, improving survival and quality of life [5–8]. The present study was conducted to assess the impact of using the upgraded system and equipment on the quality of treatment associated with the prevention of incidence of some intradialytic complications. In fact, some symptoms come about mostly during an undermanned interval in healthcare centers, so advanced facilities and artificial intelligence can take care of some functions in this condition in the dialysis center. The proposed method in this study is integrating the chair and hemodialysis machine to perform activities such as positioning, measuring weight, and using accessories along with the chair that physical activity can be performed by patients, which directly affects blood pressure and relieves some intradialytic complications, thereby improving the quality of treatment [9, 10].

## 2. Intradialytic Complications

Each patient undergoes dialysis three times a week on average of three to four hours once a time. As noted, the patients are threatened during dialysis by various complications. Despite decades of experience, there is still plenty of ongoing research to identify the causes of HD symptoms. Some researchers have focused on the recognition of modifiable predictors of intradialytic HD-related symptoms. According to clinical trials, hypotension is the most common complication occurring in dialysis sessions with symptoms such as dizziness, fatigue, and nausea [11–15] (Figures 1 and 2). One of the analyzed research studies in 2014 (44,801 HD treatment sessions with a number of 1,137 patients) showed 75.1% hypotension occurrence [16]. Another research in the sub-Saharan African health system in 2012 [17] investigated the acute complications of 1,000 HD sessions by the number of 129 patients with 25% hypotension and 22% muscular cramps. Kidney Disease Outcomes Quality Initiative (KDOQI) and European Best Practice Guidelines (EBPG) both specified the same range for hypotension as a decrease in systolic blood pressure of at least 20 mmHg [18, 19]. Occasionally, hypotension may occur due to human errors, such as low accuracy in weight measurement prior to dialysis and improper dialysis device programming in case of excessive dehydration of the patient [20]. A drop in blood pressure will lead to clotting of the patient's blood, and the dialysis process will not function properly and suitability will be reduced. Intradialytic hypotension in the long term increases the rate of cardiovascular side effects, hospitalization, and mortality [21, 22]. Preventive remedies are mainly carried out by clinicians to overcome and control the blood pressure like adjusting the dialysis fluid sodium, reducing blood flow, lowering dialysate temperature, and turning the patient position to Trendelenburg on the chair [11, 23–27]. During dialysis, a large amount of fluid is removed from the body. The circulatory system compensates for the outflow of this fluid from the body, which tightens the arteries of the muscles, especially the muscles of the arm and legs, and the blood flow to these areas decreases. Consequently, muscles become deficient in nutrition and blood supply and gradually become leaner and weaker, resulting in increased fatigue and muscle cramps. More research is agreed on the drop in blood pressure because a large amount of fluid is removed in a session [28]. Another side effect of hemodialysis that a patient may experience during dialysis is nausea and vomiting, which may cause stress and anxiety to the patient and, on the other hand, can lead to early cessation of dialysis, which is undesirable, and the adequacy of dialysis can be affected. In the majority of cases, nausea and vomiting are associated with a decrease in blood pressure [29]. The main reasons for HD complications can be divided into results from common dialysis methods, mechanical, and the advent of continuous or incomplete purification of toxins which directly affect the quality of treatment. As reported by other researchers, pharmacological therapeutic strategies may lead to different types of drug interaction or growth of toxicity in the patient's blood since their low glomerular filtration rate [30, 31].

## 3. Dialysis Dose

Dialysis adequacy is the measurement of the quality of hemodialysis treatment delivered in a session. Generally, the adequacy of dialysis is quantified by the comparison between urea distribution volume before and after blood purification. A higher reduction of urea volume in the dialysis session means how much treatment delivered was efficient. Assessment of dialysis adequacy is a crucial parameter in hemodialysis treatment which affects directly on patient morbidity and mortality [1, 32]. In the National Cooperative Dialysis Study (NCDS), research was done about the influence of the low adequacy of dialysis on chronic kidney disease (CKD) morbidity and mortality. The consequences showed substantial growth in hospitalization and incomplete treatment [33, 34]. As expected, an increase in the median dose of dialysis from 1988 to 1991 resulted in a reduction in mortality ratio from 22.8% to 9.1% (Figure 3) [35]. Other retrospective studies about the impact of dialysis adequacy on mortality in 2002 by Port et al. investigated the information of at least 4500 CKD patients treated by hemodialysis [36]. Patients were categorized based on their body weight into three types (small, medium, and large) to analyze separately the relation between adequacy and mortality ratio (Figure 4). In all types, increased adequacy leads to death rates reduction. Renal replacement therapy focused on removing urea and creatinine waste products that exist in blood during kidneys function failure. Urea distribution volume is an element utilized for dialysis dose calculation by the term Kt/V_urea_ or URR that the former is the most convenient and common index which describes the fraction of body water purified of urea during each session [35]. Although more research considered specifying the standard values of Kt/V, the significant issue is checking whether the ordered adequacy has been delivered. Most of the time, variation between the ordered and delivered dialysis adequacy is substantial [37–39].

Comparison of the prescribed dialysis dose with the actual dose delivered during the HD session to the patient can provide valuable facts or details about apparatus, systems, and blood access operation. Essentially, both prescribed and delivered adequacies should be agreed otherwise. Functionality should be noticed to deal with disagreement (Table 1) [40]. According to Table 1, prescription urea clearance can be achieved in dialysis sessions when the clinician team makes an effort to deliver the treatment efficiently by regular monitoring and controlling the HD treatment, but the increasing number of hemodialysis patients may potentially make it more complicated to provide optimal care in a medical center. Therefore, the existence of developed equipment can play a prominent role in accessing satisfactory results such as the prescribed dialysis doses and high-quality treatment.

## 4. Dialysis Dose Determination

URR, formal urea kinetic modeling (FUKM), formal single-pool urea kinetics, and online clearance monitoring (OCM) are the acceptable procedures for dialysis dose calculation. URR is a straightforward and common method in urea clearance calculation. Unlike other methods, in the URR method, the calculations have low accuracy due to the neglect of urea removal by ultrafiltration. The higher the ultrafiltration volume (UFV) removed during HD treatment, the unrealistic results are calculated for dialysis quality in this method [41, 42]. FUKM is the most precise and complex method of determination of Kt/V [43, 44]. The FUKM method requires accurate measurement of BUN concentration in the first dialysis session of the week, body weight of the patient earlier than and after the first dialysis session, urea concentration before the second dialysis session, the actual effective treatment time, and the effective urea clearance of the dialyzer as measured at the dialysis center [45]. The main disadvantage of the FUKM method is the logistical aspect. In this method, in dialysis centers, measurement of parameters such as the effective urea clearance of the dialyzer in clinical practice is so difficult. Due to the listed disadvantages of the FUKM method, the best alternative is the calculation of Kt/V with the formula presented by J.T. Daugirdas, which is also based on the analysis of blood samples [46].

(1) $$\begin{array}{c} \frac{\mathrm{Kt}}{\mathrm{Vsp}}=-\ln\left(R-0.008*t\right)+\left(4-3.5*R\right)*\frac{\mathrm{Uf}}{W}, \end{array}$$

where *R* is the correlation between blood urea nitrogen before and after dialysis, *t* denotes the time duration of detoxification in hours, *Uf* indicates patient fluid removal volume in liters during dialysis, and *W* represents patient weight after dialysis in kg.

The use of patient urea distribution volume caused by ultrafiltration and body weight in the proposed formula to determine the values of Kt/V has significantly increased the accuracy of dialysis adequacy calculations in the standard range for Kt/V values [47, 48] in comparison with the URR method.

By online clearance monitoring provided in hemodialysis care therapy systems, intradialytic measurements like the effective urea clearance (K), the total cleared blood water volume (Kt), and adequacy of dialysis (Kt/V) can be achieved automatically which does not require additional costs and most significantly patient's urea/blood sample for dialysis dose determination during hemodialysis treatment. Although single-pool Kt/V (spKt/V) is the most accurate measurement method of dialysis efficiency, the OCM has the same outcome for adequacy calculation [45].

## 5. Online Clearance Monitoring (OCM)

To access a low-cost and accessible way to monitor regularly the quality of dialysis delivered to the patient in dialysis centers, it was necessary to change the conventional methods. The best alternative to urea/blood sample purification analysis is the use of positively charged sodium ions. Although they differ in terms of size and electrical charge, both particles exhibit comparable diffusion profiles across a synthetic dialysis membrane [45]. The change in sodium concentration in the dialysis fluid is measured by sensors built into the dialysis machine. According to the similar diffusion properties in sodium ions and urea through the dialyzer membrane, urea removal and effective dialysis time can be achieved and utilized in the calculation of dialysis adequacy [49]. Dialysis dose value can be calculated by division of the total cleared blood water volume (Kt) by the urea distribution volume (V), which should be entered manually by the clinicians in the center for an individual patient. Anthropometric formulas developed by Watson [50] (2), Hume-Weyers [51] (3), and Mellits-Cheek [52] are the simplest methods of calculating urea distribution volume based on body weight, height, age, and gender.

(2) $$\begin{array}{c} \text{Male}:{\text{V}}_{\text{urea}}=2.447-\left(0.09516*\text{age}\right)+\left(0.1074*\text{height}\right)+\left(0.3362*\text{weight}\right),\\ \text{Female}:{\text{V}}_{\text{urea}}=-2.097+\left(0.1069*\text{height}\right)+\left(0.2466*\text{weight}\right), \end{array}$$

(3) $$\begin{array}{c} \text{Male}:{\text{V}}_{\text{urea}}=\left(0.194786*\text{height}\right)+\left(0.296785*\text{weight}\right)-14.012934,\\ \text{Female}:{\text{V}}_{\text{urea}}=\left(0.34454*\text{height}\right)+\left(0.183809*\text{weight}\right)-35.270121. \end{array}$$

OCM and conventional methods for the Kt/V measurement are compared by different effective factors (Table 2). It offers many advantages in using OCM to measure the dialysis dose.

## 6. Discussion

One of the most important issues for dialysis patients is maintaining proper conditions during and after dialysis. Therefore, one of the important aims of nursing care is to identify and implement comfort criteria. In most cases, nurses are unaware of the vital signs and adverse effects mentioned for patients during dialysis because they are affected by many factors. Providing appropriate care and attention to the patient's vital signs at all times while undergoing dialysis greatly enhances the effectiveness of dialysis. Performing these tasks at a dialysis center where multiple patients are being treated concurrently will often be challenging and an integrated and efficient system is necessary to ensure the automatic tracking and control of some of these tasks. An intelligent system that can take some nurse care responsibilities and choose proper intervention strategies in critical conditions improves the quality of treatment sessions. As noted, this study intended to focus on nonpharmacological interventions for preventing acute HD complications to achieve the preferred clinical outcome. The most efficient preventive strategies for hypotension, which is a common complication associated with dizziness, nausea, vomiting, headaches, or muscle cramps [53], are sodium profiling [54], reducing dialysate temperature [55], reducing ultrafiltration rate [56], changing the patient position to Trendelenburg [57], and intradialytic exercising [58]. Among these intervention strategies, sodium profiling has not concurred on whether it is useful in preventing hypotension occurrence [18]. Cooling dialysate has been shown as a safe preventive method, but its range should be noticed. Another meta-analysis defined that the use of low-temperature dialysate reduces the rate of hypotension by 70% and increases minimum arterial pressure by 12 mmHg [26]. Intradialytic exercise greatly impacts the improvement of health-related quality of life, cardiovascular outcomes, and dialysis adequacy [59–61]. Therefore, regular exercise during dialysis acts as a beneficial intervention to inhibit cardiovascular complications such as hypotension. In addition, when the patient is exercising during a muscle cramp, the muscles are diluted and perfusion increased; then, muscle blood flow that is decreased by ultrafiltration is compensated [62]. Overall, hypotension and associated side effects reduce treatment effectiveness among patients, and their blood pressure needs to be monitored by clinicians on a regular basis, which means taking extra nurses to cope with the increased workload, thus rising treatment costs [63, 64]. Monitoring vital sign parameters during HD treatments assist staff nurse to assess the general condition of a patient and take a proper strategy intervention to overcome progressing acute HD complications if it is required. The intelligent system consists of integration between the chair and HD machine in a dialysis center which is able to monitor and measure essential parameters automatically, optimize the management of treatment, and enhance the quality of care (Figures 5 and 6). The ability to perform the strategies intervention based on the data measurement is the most important characteristic of this system in comparison with research that just provides an intelligent system to predict the hypotension occurrence in HD sessions based on patient databases [65]. The principle of this system is measuring the weight (slave) and blood pressure (master). Correct weight measurement defines the proper UFV for patients during dialysis to achieve dry weight. This type of measurement reduces the risk of specified inaccurate predialysis weight by human error and an incorrect set of UFV. On the other hand, access to the patient's weight and its variations in the OCM method, in addition to updating the clearance, and nurses can be informed of how much dehydration needs to be manually adjusted, if necessary, before dialysis is completed. These continuously automatic measurements can prevent the progress of adverse complications like hypotension if preventive remedies perform on time. According to research about exercising and its beneficial outcomes on quality of treatment [66,67], the chair is equipped for aerobic exercise during dialysis (Figure 7). An original study in 2018 investigated the beneficial clinical outcomes of combination and aerobic exercises by stationary bike during dialysis with improvements in sleep quality and physical activity [68].

## 7. Conclusion

Over the past decade, efforts focused on reducing the costs of healthcare while improving access to the healthcare system and ensuring high-quality outcomes. Finding strategies to fulfill patient demands at all levels of care is crucial to improving the treatments' system functionality. Although some studies analyze the procedures of HD treatment with more beneficial suggestions, facilities were out of consideration which has a substantial effect on the quality of treatment. This study focused on facilities upgrade to enhance the quality of HD treatment by reducing clinician workload and helping the staff nurse prevent the progress of acute HD complications. Integration of the chair (slave) and HD machine (master) provides the intelligent system with the ability of automatic intervention strategies performing in critical conditions to prevent the occurrence of intradialytic complications and enhance the quality of treatment. Decision-making by the intelligent system based on gathered information and predefined instructions is a fundamental aspect of this method. This technique provides valid and reliable nonpharmacological interventions against progressing the HD side effects. Reducing dialysis temperature, reducing ultrafiltration rate, and changing the position to Trendelenburg are the functions when low blood pressure is diagnosed by master. Body weight is measured regularly by the slave and sent to the master for setting the proper UFV and dialysis dose calculation in the OCM method. In addition, intradialytic exercises by the slave equipped with special accessories have a substantial benefit in high-quality treatment.

## Figures and Tables

**Figure 1:** Prevalence of commonly reported symptoms in hemodialysis patients. NV, nausea and vomiting; DR, dialyzer reaction; DDS, dialysis disequilibrium syndrome [13].

**Figure 2:** Prevalence of intradialytic complications at the dialysis treatment session [14].

**Figure 3:** Dialysis patient's mortality reduction by increasing dialysis dose per year [35].

**Figure 4:** Diagram slopes defining the reduction of death rates correlated to increased adequacy for all types of body weight [36].

**Figure 5:** Making an artificial intelligence by connecting the chair and HD machine to deliver high-quality treatment by helping clinicians in some essential tasks; this connection (BUS) is controlled by the master (HD machine) based on predefined instructions.

**Figure 6:** Strategies aimed at controlling the connection by master (HD machine). SBP, systolic blood pressure; DBP, diastolic blood pressure; LBP, low blood pressure; BP, blood pressure; TP, Trendelenburg position; UF, ultrafiltration; CPR, cardiopulmonary resuscitation.

**Figure 7:** Movement parts of the chair proper for exercising in dialysis duration; patients push it back and forward by feet.

**Table 1:** The most common reasons for dialysis dose being less than specified urea clearance [41].

Patient-related factors	Staff-related factors	Mechanically related factors
Inadequate effective dialysis treatment session	BSR less than specified during entire dialysis time because of slow increase to specified BSR, hypotension, gradual decrease of BSR at end of dialysis	Inaccurate calibration of the blood pump

Insufficient effective bloodstream rate (BSR)	Incorrect set of dialysate flow rate	Inaccurate calibration of dialysate flow

1. Recirculation	Utilize dialyzer with inappropriate clearance	Coagulating of dialyzer fibers and “channeling”
2. Inadequate arterial bloodstream in access		
3. Utilize the catheter with bloodstream restriction		

**Table 2:** The comparison of OCM and the conventional methods for the Kt/V measurement [45].

The conventional procedure today	Aspects	5008 with OCM option
Blood samples (expensive)	Kt/v ≥ 1.2,…,1.8	Dialysate; *k* and *t* (no additional costs)
Once a month/quarterly	Frequency	In every session
Retrospective	Control	Continuous, online
Staff, syringes, lab time, cost, and energy	Effort	None
6–8%	Accuracy of k	6%
Inconvenient	Handling	Automatic
Unpractical and uncommon	Quality assurance	Standard!

## Data Availability

The data used to support the findings of this study are included within the article.
